# Pyroptosis-Related Genes as Markers for Identifying Prognosis and Microenvironment in Low-Grade Glioma

**DOI:** 10.1155/2023/6603151

**Published:** 2023-02-11

**Authors:** Jinkun Han, Yajun Jing, Peng Sun

**Affiliations:** Department of Neurosurgery, The Affiliated Hospital of Qingdao University, Qingdao 266005, China

## Abstract

Low-grade glioma (LGG) is one of the most common brain tumors and often develops into the worst glioblastoma (GBM). Pyroptosis is related to inflammation and immunization. It has been demonstrated to influence the progression of a variety of cancers. However, the value of pyrosis-related genes (PRGs) in LGG remains unclear. Public TCGA-LGG data are used to analyze the differential expression and genetic variation of PRGs in LGG. Subsequently, this paper identifies pyroptosis-related subtypes and constructs prognostic models. This paper analyzes the expression and function of selected CASP5 in LGG and constructs a ceRNA regulatory network. Final CASP5-related immune infiltration analysis and methylation analysis are performed. Most PRGs are differentially expressed and altered in LGG. Subtypes and prognostic models based on PRGs not only have good functions but also have a great connection with immune infiltration. Enrichment analysis of PRGs with prognostic value of LGG also shows functions correlated mainly with immunity and inflammation. CASP5 is significantly differentially expressed in different grades of gliomas and different prognoses. Despite fewer mutations, CASP5 has a clear correlation for both immune cells and immune checkpoint molecules in the LGG microenvironment. Its methylation may also have a role in the prognosis of LGG. This paper shows the association of pyrosis-related subtypes, prognostic models, and genes, with immune infiltration.

## 1. Introduction

Diffuse low- and intermediate-grade gliomas constitute low-grade glioma (LGG, World Health Organization (WHO) grades II and III), including astrocytomas, oligodendrogliomas, and oligoastrocytomas [1, 2]. Compared with benign WHO I glioma, WHO II and III gliomas are incurable by surgical resection and often eventually develop into glioblastoma [3, 4]. Surgery and adjuvant therapy (including radiotherapy and chemotherapy) are the basic strategies for the treatment of LGG, which has also been demonstrated in many studies to prolong the survival time of patients with LGG [5–7]. Due to the variability of tumors, pathological diagnosis cannot accurately predict prognosis [8]. Clinical decision-making for LGG now relies more on genetic typing, which is also recommended in glioma classification.

Pyroptosis is a programmed cell death (PCD) characterized by the release of proinflammatory mediators and the induction of an inflammatory response [9]. Pyroptosis is usually initiated by caspase (CASP) family proteases and is performed by gasdermin (GSDM) proteins [10]. As cell death, pyroptosis naturally plays a role in inhibiting tumor progression. Recent studies have also found that pathways and inflammatory mediators involved in pyroptosis are associated with drug resistance of tumors. In fact, much evidence exists that has demonstrated the important role of pyroptosis in a variety of cancers. However, the role of pyroptosis-related genes (PRGs) in LGG remains to some extent unknown.

Since representing tumor and surrounding stromal cells, the tumor microenvironment (TME) has tumor-specific characteristics, especially immune infiltration. The immune microenvironment infiltrated by different immune cells can promote the therapeutic resistance of tumor invasion through immunosuppression. So, immunotherapy can inhibit tumor progression by enhancing the immune system's response to tumor cells. This requires more biomarkers to characterize the prognosis and microenvironment of tumors. We start from the analysis of the LGG data from TCGA and explored the significance and function of pyroptosis-related genes in LGG by the bioinformatics analysis.

The remainder of this paper is organized as follows.  Section 2 presents the construction of the pyroptosis-related prognostic model.  Section 3 provides the experimental result and Section 4 illustrates data analysis and result discussion. Finally, the conclusion of this study and some future recommendations are given in Section 5.

## 2. Construction of the Pyroptosis-Related Prognostic Model

The paper downloads information about the LGG samples as the tumor group using The Cancer Genome Atlas (TCGA). Because TCGA lacks the corresponding normal samples, the paper obtains brain samples as normal samples at Genotype-Tissue Expression (GTEx, https://gtexportal.org/home/). We use R to make statistical analysis and visualize with R package ggplot2. 32 PRGs are obtained from prior reviews, which have described and analyzed the members of PRGs in their studies. We use the integrated database Gene Set Cancer Analysis (GSCA) to check the other information about TCGA-LGG, including the mutation frequency, waterfall plot, and the correlation between immune cell type and GSVA score of PRGs. We use the R package ConsensusClusterPlus for consistency analysis to the RNA-sequencing (RNA-seq) data from TCGA. Then, we use the R package pheatmap for clustering heatmaps and retained PRGs with standard deviation (SD) >0.1. SIGLEC15, TIGIT, CD274, HAVCR2, PDCD1, CTLA4, LAG3, and PDCD1LG2 are selected to be immune-checkpoint-relevant transcripts. We extract transcripts of immune-checkpoint-relevant 8 genes, SIGLEC15, TIGIT, CD274, HAVCR2, PDCD1, CTLA4, LAG3, and PDCD1LG2, to visualize the differential expressions among the 3 LGG subgroups, using R package ggplot2. With the same visualization methods, we utilize the R package immunedeconv which integrates many kinds of algorithms, including TIMER, to make immune infiltration estimations for 3 LGG subtypes. We use the one-class logistic regression (OCLR) algorithm constructed by Malta to calculate mRNAsi, based on the characteristics of 11774 genes' expression profile obtained from TCGA. According to Spearman correlation, we subtracted the minimum value and divide it by the linear transformation of the maximum value to eventually map the dryness index to [0, 1]. Half-maximal inhibitory concentration (IC50) is an important indicator for evaluating the therapeutic response of samples. We predicted the chemotherapeutic response of temozolomide (TMZ) for LGG patients based on the Genomics of Drug Sensitivity in Cancer (GDSC, https://www.cancerrxgene.org). The prediction process is implemented by R package pRRophetic in which the LGG samples' IC50 is estimated by ridge regression. We utilized all default parameters and summarized duplicate gene expression as a mean value for statistical comparison.

We performed the log-rank tests and univariate Cox proportional hazards regression to the expression data and survival data of LGG from TCGA using R package survival and visualized ones with *p* < 0.05 by Kaplan–Meier (KM) survival curves using ggplot2. We constructed the functional network of PRGs in Metascape and identified its functional subsets and members by MCODE component. The GO and KEGG enrichment analyses are performed and visualized through R package clusterProfiler.

We use the least absolute shrinkage and selection operator (LASSO) regression algorithm to perform feature selection on data of TCGA-LGG with the R package glmnet. During the development of the regression model, we screened the factors and reduced overfitting by forcefully changing some coefficients to zero. The log-rank is used to test survival differences in KM. Subsequently, we extracted the LGG data from CGGA (https://www.cgga.org.cn/index.jsp) to validate the constructed prognostic model. The Spearman's correlation analysis is used to describe the correlation between the risk scores and the different immune cell abundances derived by applying the TIMER algorithm.

In the analysis of tumor mutation burden (TMB) and microsatellite instability (MSI), we perform the Spearman correlation analysis to discover PRGs' correlations with them. We downloaded and merged mRNA expression data and drug sensitivity data from GDSC. By performing the Pearson correlation analysis, we obtained the correlation between the IC50 of the top 30 drugs and the PRG expression to make the bubble plot.

We search for differential expression of CASP5 between tumor and normal samples in the data on different tumors from TCGA at TIMER, a website related to immune infiltration. Afterward, we ranked the RNA expression profiles from TCGA-LGG according to the expression values of CASP5. We selected half of the patients with high CASP5 expression values for GSEA enrichment analysis and synthesized the curves of the top 7 hallmarks. We find the data about the distribution of CASP5 expression and the corresponding types of copy number value (CNV) in LGG in cBioportal and visualized their correlation by R software.

We perform prediction and intersection of target miRNAs bound to CASP5 in ENCORI and miRWalk, respectively. The correlation between 15 miRNAs and LGG is calculated by the processing of TCGA-LGG data through R software and then we screened the rest genes using the correlation with CASP5. Eventually, we obtain five miRNAs, hsa-miR-16-5p, hsa-miR-15b-5p, hsa-miR-424-5p, hsa-miR-503-5p, and hsa-miR-3690. ENCORI and LncBase-Predicted v2 are used to predict lncRNA targets that bind to miRNAs. The results of each miRNA in both websites are intersected, and a total of 63 lncRNAs corresponding to the 5 miRNAs are finally found. We construct the lnRNA-miRNA-mRNA triple regulatory network in Cytoscape and obtained a subnetwork composed of 11 hub genes with the EPC algorithm in CytoHubba, a Cytoscape plug-in. We screen 3 lncRNAs which are of prognostic value and differentially distributed between normal and LGG samples by processing data from TCGA-LGG and GTEx-brain using R software. We acquire lncRNA sequences with LNCipedia and performed cellular localization in lncLocator. The TCGA-LGG data are processed with R software to explore the correlation of the selected MCM3AP-AS1 with other molecules.

We divide LGG patients into 2 groups using the expression of CASP5 by processing the data from TCGA-LGG. We investigate the expression differences of 3 methyltransferase genes and 5 DNA repair genes between the CASP5_high group and the CASP5_low-group. We assess the methylation level of CASP5 in LGG and normal tissue in DiseaseMeth 2.0, the human disease methylation database. We find relevant methylation sites on the CASP5 sequence in MEXPRESS. MethSurv is used to evaluate the scattering of different CpG islands about CASP5.

## 3. The Experimental Results

### 3.1. Landscape of Genetic Variation of PRG in LGG

We first explore the differential expression of PRGs in normal and LGG samples. Except for PJVK, the other 31 genes are all upregulated or downregulated in LGG, as shown in Figure 1(a). Accurately, the expressions of GSDMB, ELANE, NLRP2, and IL6 are decreased in LGG, and the expression of the remaining PRGs is increased. In LGG, the frequency of mutation in NLRP2 is the highest, reaching 17%, and all missense mutations, as shown in Figure 1(b). The top 10 genes are listed, as shown in Figure 1(c).

The types of copy number variation (CNV) of PRGs in LGG are different. For example, there is mainly deletion in NLRP2 and CASP9, but mainly amplification in ELANE and GSDME, as shown in Figure 1(d). We also discover the correlation between gene expression and CNV. The results showed that the expression of CASP3, CASP6, NOD1, GSDME, SCA11, CASP9, GSDMC, CASP8, TIRAP, ELANE, IL6, NLRP2, and PLCG1 confirmed a significant positive correlation with CNV (S1). We also calculate gene set expression (GSVA) score and find that of PRGs are mainly significantly positively correlated with macrophages and negatively correlated with naive CD8+ T cell (S2).

### 3.2. PRGs-Based LGG Subtype

In order to explore the relationship between the expression of PRGs and LGG subtypes, we use consensus clustering analysis to classify the LGG patients. By increasing the clustering variable (*k*) from 2 to 10, the most appropriate number of classifications is observed when *k* = 3, as shown in Figure 2(a). The heatmap demonstrates the expression of PRGs in the 3 groups (S.3A). We calculated the prognosis of the three clusters and found that C3 had a significantly worse prognosis compared with C1 and C2, as shown in Figure 2(b). We compare the expression of eight immune checkpoint genes for three clusters. The results show that the expression levels of these genes in G3 are all the highest, as shown in Figure 2(c). The same situation is also observed by immune cell score, except for CD8+ T cell, as shown in Figure 2(d). Myeloid dendritic cells are the highest proportion of the six immune cells. Considering that 3 types may reveal that a worse prognosis in LGG is associated with the acquisition of stem-like features, we apply OCLR to find the highest score in G1 but the lowest one in G3, as shown in Figure 2(e). Finally, we predict the response of the three classes of LGG to treatment with TMZ and found that the IC50 of G3 is the lowest. Moreover, we explore the differential expression of 32 PRGs among 3 clusters, as shown in Figure 2(f). Except for SCAF11 and GPX4, we find that there are differential expressions of all other PRGs among 3 clusters. Most of the PRGs had the highest expression in G3.

### 3.3. Functional Enrichment Analysis of Prognostically Relevant PRGs in LGG

By the univariate COX regression, we find 18 genes with prognostic value in PRGs, and the KM survival curves are shown in Figure 3. High expressions of all 18 PRGs except for CASP9 and GSDMC are associated with a worse prognosis of LGG. To understand the action pathway of this part of PRGs on LGG, we perform functional enrichment analysis on the genes with prognostic value. Top biological process (BP) is the regulation of cysteine-type endopeptidase activity, response to lipopolysaccharide, and response to molecule of bacterial origin. Cellular component (CC) is mainly enriched in the cytosolic part, and the major molecular function (MF) is cysteine-type endopeptidase activity and cysteine-type peptidase activity. We perform the KEGG enrichment analysis and found that the most relevant KEGG pathways of PRGs with prognostic value are NOD-like receptor signaling pathway, legionellosis, and pathogenic *Escherichia coli* infection. We synthesize their enrichment analysis in Metascape and constructed functional networks, where the subsets and its members of the network involved the two most significant functions. The associated *P* value network shows NOD-like receptor signaling pathway as the most significant functional term (S.4A), which participated in immune system. Interestingly, the circle shows that NLRP6, NLRP1, and GSDMD only involve this term in the top 20 KEGG pathways (S.4B). Eventually, we visualized the expression correlation of 18 PRGs with prognostic value. The results showed that there are often associations between every 2 PRGs (S.4C). Figure 3 displays the KM curves of PRGs with the prognostic value in LGG.  Figure 4 shows functional enrichment analysis of prognostically relevant PRGs.

### 3.4. Construction of a Prognostic PRG Model

By forcing the regression coefficients of some members of the 32 PRGs to be reduced to zero and applying cross-validation to avoid overfitting, we construct the stable prognostic model. We finally identify and screen 10 genes by the LASSO Cox regression analysis (S. 5A, 5B). Risk score = (0.079)*∗*PRKACA + (−0.4102)*∗*CASP9 + (0.8144)*∗*PLCG1 + (0.5394)*∗*CASP4 + (0.0591)*∗*CASP3 + (0.1184)*∗*IL8 + (0.1916)*∗*CASP8 + (−0.1366)*∗*GSDMC + (−0.2229)*∗*CASP5 + (0.0314)*∗*CASP1. We divide the LGG patients into two groups according to the risk score and explore their prognostic difference, as shown in Figure 5(a). The results demonstrated that patients with high scores had a shorter survival time, as shown in Figure 5(b). The AUC of ROC curves at 1 year, 3 years, and 5 years are 0.885, 0.875, and 0.761, respectively, as shown in Figure 5(c). In the validated data from CGGA-LGG, there is also a significant survival difference between patients in the high-risk and low-risk groups (S. 5C, 5D). The ROC curves also validated the predictive value of the model for survival in patients with LGG (S. 5E). The combined diagnosis value of these PRGs is also higher than every member alone as shown in Figures 5(d) and 5(e). We perform TIMER immune scoring on the prognostic model and find that the risk score is significantly correlated with B cell, CD4+ T cell, neutrophil, macrophage, and dendritic cell, as shown in Figure 5(f).

### 3.5. MSI, TMB, and Drug Susceptibility Associated with PRGs

Tumor mutation burden (TMB) and microsatellite instability (MSI) have received increasing attention as indicators that can predict the efficacy of immunotherapy. We explore the correlation between the expression of PRGs of prognostic models in LGG and TMB and MSI to identify whether they could be used as markers for immunotherapeutic drug screening. The results demonstrated a negative correlation between the expression of CASP1 and MSI (*p*=0.049, cor = −0.09) and a negative correlation between the expression of PLCG1 and MSI (*p*=0.001, cor = 0.15). GSDMC (*p* = 8.49*E* − 06c, cor = −0.2) is revealed to have a negative relationship with TMB, which is positively correlated with the expression of other members of the prognostic models except for CASP9. To search for possible drugs, we explored the expression of these 10 genes in relation to the sensitivity of existing drugs.  Figure 6 shows the correlation of PRGs expression in LGG with TMB, MSI, and sensitivity of existing drugs.

### 3.6. Building Relevant Nomogram

Considering the possible response effect of clinical factors on LGG, we construct a nomogram involving clinical factors and PRGs expression to predict overall survival. The univariate and multivariate analyses screened out multiple independent factors, as shown in Figures 7(a) and 7(b). The factors for the best nomogram of the final combination include grade and the expression of CASP9, CASP5, and PLCG1, as shown in Figure 7(c). However, this nomogram is shown to well predict the 1-year, 3-year, and 5-year overall survival rate of LGG patients, as shown in Figure 7(d).

### 3.7. Expression, Variation, and Functional Analysis of CASP5 in LGG

The conversion of LGG to GBM is thought to be one of the reasons for the poor outcome of LGG. We explored the correlation between the expressions of nomogram members in glioma. Only CASP5 is revealed to distinguish 3 grades of gliomas, as shown in Figure 8(a). Therefore, we perform further analysis around CASP5. Similar to LGG, CASP5 is also significantly highly expressed in esophageal carcinoma (ESCA), head and neck squamous cell carcinoma (HNSC), and uterine corpus endometrial carcinoma (UCEC) (S. 6A). To further search for functions associated with CASP5, we performed GSEA enrichment analysis on patients with high expression of CASP5 in TCGA-LGG. The significant hallmarks are a complement, allograft rejection, as shown in Figure 8(b). The set containing the 200 genes most correlated with the expression of CASP5 is shown to be concentrated in neutrophil activation and neutrophil degranulation in BP, secretory granule membrane and MHC class II protein complex in CC, MHC protein complex binding, and MHC class II protein complex binding in MF by the GO enrichment analysis (S. 6B). The KEGG pathways are mainly focused on *Staphylococcus aureus* infection, leishmaniasis, and phagosome (S. 6C). The heatmap shows the expression distribution of the top 15 genes in KEGG-LGG (S. 6D).

We explored the changes of the CASP5 expression among different subgroups of LGG. The expression of CASP5 in astrocytoma is significantly higher than that in oligoastrocytoma and oligodendroglioma, as shown in Figure 8(c). Compared with patients belonging to complete response (CR), partial response (PR), and stable disease (SD), the expression of CASP5 is significantly higher in progressive disease (PD) of LGG, as shown in Figure 8(d). The LGG patients who have wild IDH status or noncodeletion of 1p/19q both have higher CASP5 expression, as shown in Figures 8(e) and 8(f). The expression of CASP5 is associated with the mutation of LGG-related signature genes. We found that CASP5 is highly expressed in patients with mutant EGFR, as shown in Figure 8(g), and the same in patients with mutant P53, as shown in Figure 8(h). Finally, we also explore the mutation of CASP5 in LGG. The alteration frequency of CASP5 in LGG is low (S. 6E). Although CASP5 expression is higher in patients with shallow deletion (S. 6F), it is not found to have a significant correlation with copy number value (S. 6G).

### 3.8. Construction of CASP5-Related ceRNA Network

By ENCORI and miRWalk, we predict 5 miRNAs that regulate CASP5, which had not only prognosis value but also correlated expression with CASP5's (S. 7A, 7B). Afterward, we identify a total of 63 lncRNAs associated with these 5 miRNAs by ENCORI and lncBase-Predicted v2. To explore the molecular regulatory mechanism of CASP5, we construct a lncRNA-miRNA-mRNA regulatory network and selected a subnetwork including 11 hub genes by EPC in Cytoscape, as shown in Figures 9(a) and 9(b). We find AGAP2-AS1, LINC00665, and MCM3AP-AS1; all had prognostic value and were differentially expressed between LGG and normal samples among seven hub lncRNA-related genes, as shown in Figures 9(c) and 9(d). Considering that cellular localization determines the underlying mechanism of the molecule, we perform subcellular localization for 3 lncRNAs. The results show that MCM3AP-AS1 is mainly located in the cytoplasm, but AGAP2-AS1 and LINC00665 are mainly distributed in exosome and cytosol, as shown in Figure 9(e). It indicates that MCM3AP-AS1 may act as a ceRNA to regulate the expression of CASP5 through hsa-miR-15b-5p/hsa-miR-424-5p/has-miR-16-5p. We discover correlations between MCM3AP-AS1 and the corresponding miRNAs and constructed ceRNA network, as shown in Figures 9(f) and 9(g).

### 3.9. Relationship between CASP5 and Immune Infiltration in LGG

Immune infiltration has received increasing attention due to its important role in tumor growth and immunotherapy. We performed immune infiltration analysis on TIMER in relation to the expression of CASP5 in LGG. We first explore the correlation of CASP5 expression with different immune cells. We found that CASP5 expression showed a significant positive correlation with all 6 immune cells, as shown in Figure 10(a). In 5 types of copy number alteration, arm-level deletion and arm-level gain are confirmed to be associated with B cell, CD4+ T cell, macrophage, neutrophil, and dendritic cell, as shown in Figure 10(b). To further validate the relationship between immune cell infiltration and CASP5 in LGG, we explored the correlation between CASP5 and the immune marker gene set of 16 immune cells. The results demonstrated that each gene set standing immune cell had members that are significantly correlated with CASP5 expression in LGG (S8). We collected 44 immune checkpoint genes and explored the association of CASP5 with them. We revealed that CASP5 expression correlates with a variety of immune checkpoint molecules (S9).

Considering that PRGs-based subtypes are also significantly associated with immune cells and immune checkpoint molecules, we explore the expression distribution of CASP5 among the three subtypes and showed that the direction of change of CASP5 among different subtypes is consistent with the direction of the change of immune checkpoint and immune cell abundance with 3 subtypes, as shown in Figure 10(c). It demonstrates that the association of PRGs-based LGG typing with immunity may be related to CASP5. We also find a high level of 6 immune cells which indicated worse 3-year, 5-year, and 8-year overall survival, as shown in Figure 10(d).

### 3.10. Relationship of CASP5 Expression with Methylation and DNA Repair in LGG

Methylation of DNA controls gene expression by regulating DNA structure, DNA stability, and the interaction between DNA and protein. We explored the effect of CASP5 expression on the expression of 3 methyltransferases and found that DNMT1 and DNMT3A are highly expressed in the CASP5_high group, as shown in Figure 11(a). The information in DiseaseMeth version 2.0 revealed that CASP5 had significantly higher methylation values in normal samples than in disease samples, as shown in Figure 11(b). In addition, we found the presence of methylation sites (cg10825847) in the sequence of CASP5, which negatively correlated with the expression of CASP5, as shown in Figure 11(d). The methylated regions associated with CASP5 are shown as a heatmap (S. 10A). We found an identical methylation site, cg10825847, which is located in the open sea region and TSS1500 region. Survival analysis showed that it is associated with a better prognosis (S. 10B). Finally, we also explored the relationship between the expression of CASP5 and DNA repair genes, and the results showed that MSH6 is highly expressed in the CASP5_high group, but PMS2 and EPCAM are opposite, as shown in Figure 11(c).

## 4. The Experimental Result Analysis

Pyroptosis has been suggested to be a form of regulated cell death (RCD) due to its dependence on the activation of inflammatory CASP and plasma membrane pores composed of GSDM protein. RCD plays an important role in removing abnormal cells and even neural development. Pyroptosis can kill infected cells and fix bacteria, which will later be killed and phagocytosed by neutrophils and macrophages. In neuroscience, pyroptosis has been found to be involved in a variety of neurological injuries, including stroke, traumatic brain injury, and brain infection. In addition, pyroptosis is also involved in the disease process of neurological diseases such as Alzheimer's disease, epilepsy, and multiple sclerosis due to the pyroptosis of neurons. The relationship between pyroptosis and cancer is complex. In addition to the anticancer effect of the pyroptosis process, the microenvironment constituted by pyroptosis molecules promotes tumor progression. In our study, we explored the impact of pyroptosis on the prognosis of LGG and identified TME associated with pyroptosis in LGG, especially the immune microenvironment. Finally, we focused on the analysis of the role of the pyroptosis-related CASP5 in LGG.

We identify 3 subtypes with significant prognostic differences by analysis of the expression profile of PRGs in LGG (*P*  <  0.0001). The progression of cancer is associated with the acquisition of stem cell-like features. Glioma stem cell is an important reason why gliomas remain resistant and eventually recur. The discordance between the OCLR score and the prognostic situation of the 3 subtypes demonstrates that the prognostic value of glioma subtypes identified by PRGs involves fewer factors of cancer stem cells. An immune microenvironment is also an important factor affecting tumor progression. Originally, antitumor immune cells are reprogramed into an immunosuppressive phenotype in the TME, which can help gliomas suppress, regulate, or even escape from the immune response. We found that the GSVA scores for the collection of PRGs are associated with a variety of immune cells in LGG. Among the 3 types associated with pyroptosis, the type with a worse prognosis is often identified with higher infiltration of immune cells by the TIMER algorithm. Immune checkpoints have recently been increasingly recognized as an important interfering target for cancer immunotherapy because they are thought to promote the immunosuppressive function of TME. For example, CTLA4 can inhibit T cell activation and promote its exhaustion, while enhancing regulatory T cell-induced immunosuppression by downregulating CD80 and CD86 on antigen-presenting cells. In our study, the expressions of 8 immune checkpoint molecules including CTLA4 are all highest in Group3. Combined with its worst prognosis and lowest temozolomide sensitivity, these reasons suggest that PRGs may alter TME by affecting immune infiltration of LGG, ultimately distinguishing different resistance and survival of the LGG patients.

Functional enrichment analysis of 18 PRGs with prognostic value in LGG showed that they mainly involved infection and inflammation. In addition to the involvement of immune function, inflammation has been suggested to induce tumor progression and angiogenesis, which is also the target of antivascular agents for gliomas. Marinari's study also demonstrated that inflammation is associated with a worse prognosis in gliomas. These results demonstrate that these 32 PRGs may play a role in the progression and prognosis of LGG.

We screen 10 PRGs with prognostic value by the LASSO regression to construct a prognostic model of LGG. The prognostic models have a satisfying predictive effect on the 1-, 3-, and 5-year survival rates of patients with LGG. The difference in median survival time between the high-risk and low-risk groups according to the risk score based on 10 PRGs is approximately 6 years. In addition to this, the great value of the combined diagnosis to LGG based on 10 PRGs indicates their potential to distinguish glioma from normal. Interestingly, we also found a significant association of 6 immune cells with a risk score based on the PRGs. However, high scores always imply an upregulation of immune cell abundance, which further demonstrates that pyroptosis affects the prognosis of LGG through immune infiltration.

MSI, as a molecular signature in cancers with deficient DNA mismatch repair, is the marker for the diagnosis and effective immune checkpoint blocking therapy in a variety of cancers. TMB has recently been shown to predict immunotherapeutic responses in a variety of tumors, also correlates with immune infiltration and cancer prognosis. High TMB frequently predicts a better prognosis after immunotherapy. Our study found multiple PRGs associated with MSI or TMB in LGG. These genes have the potential to predict the immunotherapeutic response of LGG. Subsequently, we screened PLCG1, CASP5, and CASP9 as independent prognostic factors of LGG by the Cox regression, which constituted a nomogram with glioma grade. Calibration plots show that nomograms can predict survival at 3 years and 5 years relatively well compared to ideal models.

Since CASP5 is found to be the only pyroptosis-related gene among the individual independent prognostic factors of LGG that could distinguish grade II, III, and IV gliomas, we chose CASP5 for subsequent analysis. CASP5 is an inflammatory protease involved in inflammatory and cell death processes, which involves a cascade of enzymatic reactions mediated by multiple members of the CASP family. CASP5 has a role in a variety of diseases such as arthritis, psoriasis, and cancer. We also find that CASP5 had high expression similar to LGG in ESCA, HNSC, and UCEC in our study. However, the mutation frequency of CASP5 is low, which indicates that the role of CASP5 in LGG is less associated with mutations. This is the same conclusion as the previous study. We perform the GSEA enrichment analysis on the highly expressed cohort, while the GO and KEGG enrichment analysis on the related genes. The results show multiple functions regarding immunity and inflammation such as complement, neutrophil activation, MHC class II protein complex, MHC protein complex binding, and *Staphylococcus aureus* infection. These imply the correlation of CASP5-involved pyroptosis with a variety of biological processes. In addition to differential expression in different pathological types, CASP5 is also significantly highly expressed in PD, which also confirms the abovementioned result that the LGG patients with high CASP5expression are accompanied by poor prognosis. The LGG patients with IDH mutation are generally considered to have both ATRX and TP53 mutations. IDH mutation and 1p/9q codeletion both are important factors in the poor prognosis of glioma. The significantly low expression of CASP5 in patients with IDH mutations and 1p/9q codeletion in our study indicates the relationship of CASP5 with multiple factors affecting the prognosis of LGG.

The ceRNA regulatory network is involved in the progression of a variety of cancers. In order to further explore the regulatory process of CASP5, we construct a CASP5-related ceRNA triple network in LGG. We finally find three miRNAs and one lncRNA regulating CASP5, hsa-miR-15b-5p, hsa-miR-424-5p, hsa-miR-16-5p, and MCM3AP-AS1, by prediction and screening processes including survival analysis, correlation analysis, and subcellular localization. hsa-miR-15b-5p is demonstrated to predict the LGG outcome and participate in the pathogenesis of intracerebral hemorrhage. In addition to the association of hsa-miR-424-5p with thyroid cancer, esophageal cancer, and cholangiocarcinoma, it can also be enriched in extracellular vesicles in patients with Alzheimer's disease and has diagnostic value. As for hsa-miR-16-5p, it involves research on cancer, immune disorders, and even psychosis. MCM3AP-AS1 has been shown to be involved in glioma progression and regulates angiogenesis in glioblastoma through the ceRNA axis. Our analysis revealed that it also has prognostic and regulatory value in LGG.

The immune infiltration of cancer can affect the prognosis of patients. We confirm a significant positive correlation between CASP5 expression in LGG and the abundance of all six immune cells. This is also consistent with the results of the abovementioned enrichment analysis focusing PRGs and functional analysis of CASP5-related genes. We find differential expression of CASP5 in the LGG subtypes identified by us. Combined with the prognostic difference of LGG subtypes and the prognostic impact of CASP5 on LGG, we speculate that CASP5 may be the role of immune infiltration affected by CASP5 on LGG subtypes, which needs further experimental confirmation. We subsequently also revealed the dramatic impact of the infiltration of six immune cells on the prognosis of LGG. In addition, we also demonstrate that CASP5 has different degrees of correlation with 16 immune marker gene sets and many immune checkpoints. These all imply the great potential of CASP5 in the immunotherapy of LGG. Although there is no experimental evidence, immunosuppression against CASP5 is theoretically feasible, which is similar to the current use of different immune checkpoint inhibitors in different cancers.

The DNA mismatch repair system maintains genetic stability and integrity, and we found that the LGG patients with high CASP5 expression had elevated expression of two DNA repair genes, PMS2 and EPCAM. DNA methylation plays an important role in gene regulation. We attempt to analyze the pattern of CASP5 abnormal expression in LGG by exploring DNA methylation and found CASP5 hypomethylation in LGG samples, which is consistent with the upregulation of CASP5 observed by analysis to DNA methyltransferases (DNMT1H and DNMT3A). In addition, we found that some methylation sites had significant associations with the prognosis of the HCC patients, especially cg10825847, which is validated in both databases. Its methylation is associated with a better prognosis in patients with LGG. Interestingly, all the hypermethylated sites of CASP5 fall into the open sea region. These suggest that abnormalities in methylation may be associated with the prognosis of LGG.

## 5. Conclusion

Although our study demonstrates the great potential application value of prognosis in LGG, there are still some limitations, especially the lack of experimental validation. In the future, we can experimentally analyze the mechanism of PRGs' impact to immune microenvironment in LGG. It is also necessary to explore the possibility of alleviating or even reversing the deterioration of the immune microenvironment in LGG by targeting PRGs, ultimately inhibiting the progression of LGG. Our study can serve as the first step in this encouraging process.

In summary, using public TCGA-LGG data, we construct pyroptosis-related subtypes, which may affect prognosis through differences in immune infiltration. We also construct a prognostic model for PRGs, which also showed a huge relationship with immunity. Subsequently, we focus on analyzing the function of pyroptosis-related CASP5 in LGG. We construct a potential ceRNA network of CASP5 and revealed the great impact of CASP5 on the immune microenvironment of LGG. All these imply an important role of pyroptosis in LGG, which deserves further experimental investigation.

## Figures and Tables

**Figure 1:** Expression and mutation of PRGs in LGG.

**Figure 2:** Characteristics of the 3 LGG classifications.

**Figure 3:** KM curves of PRGs with prognostic value in LGG.

**Figure 4:** Functional enrichment analysis of prognostically relevant PRGs.

**Figure 5:** The construction of the prognostic model.

**Figure 6:** Correlation of PRGs expression in LGG with TMB, MSI, and sensitivity of existing drugs.

**Figure 7:** Construction of correlated predictive nomogram.

**Figure 8:** Expression distribution of CASP5 in different subgroups.

**Figure 9:** Construction of ceRNA network.

**Figure 10:** Association of CASP5 with immune infiltration: (a) correlation between expression of CASP5 and immune cell infiltration; (b) gene copy number of CASP5 in relation to immune cells in LGG; (c) distribution of CASP5 in LGG classification; (d) KM curves analyzing the relationship between immune cell levels and overall survival in LGG.

**Figure 11:** Methylation analysis of CASP5 in LGG: (a) correlation between the expression of three methyltransferases and CASP5; (b) different distribution of methylation values between normal samples and LGG samples; (c) correlation between the expression of DNA repair genes and CASP5 expression; (d) relationship between methylation sites of CASP5 and gene expression are visualized with MEXPRESS.

## Data Availability

Publicly available datasets are analyzed in this study. The datasets analyzed during the current study are available in the following web links: GTEx, https://gtexportal.org/home/; GDSC, https://www.cancerrxgene.org; CGGA, http://www.cgga.org.cn/index.jsp; TIMER, https://cistrome.shinyapps.io/timer/; cBioportal, https://www.cbioportal.org/; ENCORI, https://starbase.sysu.edu.cn/; miRWalk, http://mirwalk.umm.uni-heidelberg.de/; LncBase Predicted v2, https://carolina.imis.athena-innovation.gr/diana_tools/web/index.php?r=lncbasev2/index-predicted; DiseaseMeth 2.0, http://bio-bigdata.hrbmu.edu.cn/diseasemeth/; MEXPRESS, https://mexpress.be/; MethSurv, https://biit.cs.ut.ee/methsurv/.
